This article has been retracted.

# MIP-1*α* Level and Its Correlation with the Risk of Left Atrial Remodeling in Patients with Atrial Fibrillation

**DOI:** 10.1155/2022/1756268

**Published:** 2022-06-24

**Authors:** Chen Bai, Qing Ye, Yichen Zhao, Yang Liu, Jiangang Wang

**Affiliations:** Department of Cardiac Surgery, Beijing Anzhen Hospital, Capital Medical University, Beijing 100029, China

## Abstract

The aim of this study is to investigate the expression level of macrophage inflammatory protein-1*α* (MIP-1*α*) in atrial fibrillation patients and its correlation with the risk of left atrial remodeling. A total of 64 atrial fibrillation patients admitted to our hospital from April 2020 to December 2021 were prospectively selected as the case group and 61 healthy subjects who received physical examination during the same period were selected as the control group. Serum MIP-1*α* level was determined by a double-antibody sandwich enzyme-linked immunosorbent assay. Serum MIP-1*α* expression levels were compared between the case and the control groups. The case group was divided into high-level and low-level groups according to the serum MIP-1*α* median. Simultaneously, the sociodemographic data, clinical data, and left atrial remodeling indexes of the patients were collected in the case group. The Pearson correlation analysis was applied to analyze the correlation between the serum MIP-1*α* level and the risk of left atrial remodeling in patients with atrial fibrillation. The serum MIP-1*α* level was significantly higher in the case group than that in the control group (*P* < 0.05), high-level group (≥2.14 pg/mL, 32 cases), and low-level group (<2.14 pg/mL, 32 cases). There were significant differences in the anteroposterior diameter, upper and lower diameter, left and right diameter of the left atrium, left atrial volume, volume index, left atrial global ejection fraction, and sphericity between the low-level and high-level groups (*P* < 0.05). The Pearson correlation analysis showed that serum MIP-1*α* level was positively correlated with the left atrial anteroposterior diameter (*r* = 0.745), left atrial left and right diameter (*r* = 0.759), left atrial upper and lower diameter (*r* = 0.810), left atrial volume (*r* = 0.837), left atrial volume index (*r* = 0.813), and left atrial sphericity (*r* = 0.785) but negatively correlated with the left atrial global ejection fraction (*r* = -0.731) (*P* < 0.05). The expression level of serum MIP-1*α* is high in atrial fibrillation patients and is associated with the risk of left atrial remodeling.

## 1. Introduction

The ectopic impulse theory of atrial fibrillation, the single-loop reentry theory, and the multiwavelet reentry theory are cornerstones for understanding the mechanisms of the occurrence and maintenance of atrial fibrillation, which increase the risk of ischemic stroke, systemic embolism, heart failure, and mortality [1]. Electrical and structural remodeling plays an important role in the pathophysiology of the development of atrial fibrillation. The early changes in atrial remodeling are usually dominated by electrical remodeling (changes in electrophysiological and ion channel characteristics), which are reversible to a certain extent. In the later stage, atrial remodeling is the main feature, which is irreversible. Atrial remodeling is associated with adverse cardiovascular events such as atrial fibrillation and heart failure, which in turn aggravate atrial remodeling, forming a vicious cycle [2]. Among atrial remodeling, left atrial remodeling is thought to be the driving force for the progression of atrial fibrillation. Therefore, it is of positive significance to seek the levels of biomarkers that can predict left atrial remodeling.

There is mounting evidence [3] that inflammatory and fibrotic cytokines are involved in atrial fibrillation and left atrial remodeling. Furthermore, inflammation, inflammation-related structural changes, and fibrosis have been implicated in atrial fibrillation development and left atrial remodeling. Macrophage inflammatory protein-1*α* (MIP-1*α*), a chemokine secreted by fibroblasts and macrophages, is involved in inflammatory responses and exerts a crucial effect on the pathogenesis of the cardiovascular disease [4]. A previous study [5] has shown that MIP-1*α* is involved in the induction of autoimmune myocarditis, which leads to the development of heart failure and increases the risk of dilated cardiomyopathy. A study [6] on circadian rhythms in cardiovascular biology and disease has confirmed that the circadian clock genes such as NR1D1 and RORC may help maintain a normal heart rhythm, and the interruption of the expression of the above circadian clock genes may affect the MIP-1*α* expression. These studies all indicate that MIP-1*α* may have an impact on the atrial structure, but the relationship between the two is not clarified. To further clarify whether MIP-1*α* is associated with left atrial remodeling, this study investigated the MIP-1*α* level and its correlation with the risk of left atrial remodeling to provide new biomarkers for the prevention and treatment of left atrial remodeling in atrial fibrillation patients.

## 2. Data and Methods

### 2.1. Clinical Baseline Data

After approval by the hospital ethics committee, 64 atrial fibrillation patients admitted to our hospital between April 2020 and December 2021 were prospectively enrolled in this study. Inclusion criteria were as follows: (1) meeting the diagnostic criteria of atrial fibrillation [7], and 12-lead ECG or 24-h dynamic ECG indicates atrial fibrillation; (2) New York Heart Association function class I-II; and (3) signing written informed consent. Exclusion criteria were as follows: (1) combined with a history of cardiac surgery; (2) combined with various valvular heart diseases and congenital heart diseases; and (3) patients with secondary atrial fibrillation due to hyperthyroidism or alcohol. Simultaneously, 61 healthy subjects who received physical examination during the same period were recruited as the control group. The serum MIP-1*α* level was measured by a double-antibody sandwich enzyme-linked immunosorbent assay. The serum MIP-1*α* expression level was compared between the case and the control groups. The case group was assigned to high-level and low-level groups according to the serum MIP-1*α* median. Simultaneously, the sociodemographic data, clinical data, and left atrial remodeling indexes of the patients were collected in the case group. The correlation between serum MIP-1*α* levels and the risk of left atrial remodeling in atrial fibrillation patients was analyzed by the Pearson correlation analysis.

### 2.2. Methods

#### 2.2.1. General Data

Information on the sex, age, body mass index, comorbidities (hypertension, diabetes, hyperlipidemia, and coronary artery disease), smoking history, duration of atrial fibrillation, type of atrial fibrillation (paroxysmal and persistent), CHA2DS2-VASC score (congestive heart failure/left ventricular dysfunction (C), hypertension (H), diabetes (D), vascular disease (V), age of 65–74 years (A), sex (female) (Sc) 1 point, age of ≥75 years (A) is 2 points), and cardiac function classification were collected.

#### 2.2.2. Determination of Serum

MIP-1*α* levels Five mL of fasting venous blood were harvested from patients of the case and control groups in the morning and maintained in a place without stirring at room temperature for 2–4 h. The blood was centrifuged at 3000 r/min for 30 min to separate and obtain serum. An automatic biochemical analyzer (Hitachi 7170A, Hitachi Co., Ltd., Tokyo, Japan) was employed to detect serum MIP-1*α* levels using a double-antibody sandwich enzyme-linked immunosorbent assay. Briefly, the standard and samples to be tested were added to the corresponding wells, followed by incubation with the detector antibody labeled with horseradish peroxidase. The plate was covered with a sealing film and incubated in a 37°C water bath for 60 min. The reaction solution was discarded and the plate was patted dry after washing, followed by incubation with the corresponding substrate at 37°C in the dark for 15 minutes. Finally, 50 *μ*L termination solution was added, and within 15 minutes, OD values at a wavelength of 450 nm were obtained using a microplate reader (Bio-Rad, Hercules, CA, USA).

#### 2.2.3. Measurement of the Left Atrial Remodeling Index

Color Doppler ultrasonography (Hubei RenXu Medical Equipment Co., Ltd., Hubei, China) was applied for cardiac examination. The patient was lying on the left side or in a supine position, breathing calmly. The left atrial diameter was measured in the parasternal left ventricular long-axis aortic root section. The left ventricular end-systolic and end-diastolic volumes were measured by recording the real-time motion trajectory of the mitral valve annulus at the apical four-chamber, two-chamber, and apical left heart long-axis views. After acquiring the apical four-chamber image in two-dimensional imaging mode, the left three-dimensional volume data were transmitted to the workstation. The rotary cutting method is adopted on the quantitative software of the processing workstation to obtain three mutually orthogonal reference planes of the left atrium and to record the left atrial volume and the left atrial volume index (left atrial volume index = left atrial volume/normalized body surface area, human normalized body surface area = 0.0061 × height (m) + 0.0124 × weight (kg) − 0.0099).

All patients underwent left atrial CT angiography: 64-slice gemstone energy spectral CT (Shanghai RanZhe Instrument Equipment Co., Ltd., Shanghai, China) was used with the following scanning parameters: tube voltage: 120 kV; tube current: 350–750 mA; slice thickness: 0.625 mm; pitch: 0.26; slice spacing: 0.625 mm; and tube rotation time: 0.35 s/circle. The patients were scanned from head to foot in the supine position. ECG signal frequency and heart rate of the patients were monitored by three ECG leads. The scanning range was from the aortic arch to the diaphragm and the left atrial images were collected. The scanned images were sent to the ADW4.4 workstation for image processing. Cardiac software was utilized to analyze the left atrial function and measure the anteroposterior diameter, upper and lower diameter, and the left and right diameter of the left atrium (the left atrial projection on the horizontal and sagittal planes could be utilized to measure the maximum value in the corresponding direction, and the maximum value of the three was applied as the approximate maximum left atrial diameter line), and the left atrial ejection fraction and left atrial sphericity were automatically calculated.

### 2.3. Quality Control

The training was unified and a unified investigation plan was determined. The inclusion and exclusion criteria were strictly implemented to ensure the objectivity and accuracy of the research data. Data were double-entered into Epidata software to ensure that all data were correct.

### 2.4. Statistical Methods

Data were analyzed using SPSS 22.0 software. Count data were expressed as *n* (%). The differences between groups were compared utilizing the *χ*^2^ test. Continuous variables that met the normal distribution were expressed as the mean ± SD and compared with the independent samples *t*-test. GraphPad Prism was applied to compare serum MIP-1*α* levels between the case and control groups. The Pearson correlation analysis was employed to analyze the correlation between the serum MIP-1*α* level and the risk of left atrial remodeling in atrial fibrillation patients. R software was used to draw a heatmap. At the *α* = 0.05 level, a value of *P* < 0.05 was considered statistically significant.

## 3. Results

### 3.1. Comparison of Serum MIP-1*α* Levels between the Case and the Control Groups

The serum MIP-1*α* level was significantly higher in the case group than that in the control group (*P* < 0.05) as shown in Figure 1; high-level group (≥2.14 pg/mL, 32 cases) and low-level group (<2.14 pg/mL, 32 cases).

### 3.2. Comparison of Clinical Data of the Case Group

The differences in age, sex, cardiac function classification, atrial fibrillation course, and type of atrial fibrillation were not statistically significant between the high-level and low-level groups (*P* > 0.05) as shown in Table 1.

### 3.3. Comparison of Left Atrial Remodeling Indexes between the Low-Level and High-Level Groups

Significant differences in the anteroposterior diameter, upper and lower diameter, left and right diameter of the left atrium, left atrial volume, volume index, left atrial global ejection fraction, and sphericity were detected between the low-level and high-level groups (*P* < 0.05) as shown in Table 2.

### 3.4. Correlation between the Serum MIP-1*α* Level and Left Atrial Remodeling Risk in Patients with Atrial Fibrillation

The Pearson correlation analysis results showed that serum MIP-1*α* level was positively correlated with the left atrial anteroposterior diameter (*r* = 0.745), left and right diameter (*r* = 0.759), left atrial upper and lower diameter (*r* = 0.810), left atrial volume (*r* = 0.837), left atrial volume index (*r* = 0.813), and left atrial sphericity (*r* = 0.785) but negatively correlated with the left atrial global ejection fraction (*r* = -0.731; *P* < 0.05) as shown in Figure 2.

## 4. Discussion

Although the pathogenesis of atrial fibrillation is still unclear, it is known that atrial structural remodeling plays an important role in the occurrence and development of atrial fibrillation. In an animal model study [8] and a clinical observational study [9], the pathophysiological characteristic changes in left atrial remodeling can lead to abnormal changes in the ultrastructure of atrial myocytes and promote myocardial fibrosis. The alterations in the left atrial structure and functional indicators were correlated with the duration of atrial fibrillation and the incidence of mural thrombosis. A molecular mechanism study has shown [10] that the occurrence of atrial fibrillation involves the activation of various regulatory mechanisms throughout the body. The increase in cytokines and infiltration of inflammatory cells cause alterations in the structure of cardiomyocytes and interstitial cells, which in turn results in structural and functional remodeling of the heart. This suggests that inflammation may exert a crucial effect on the risk of left atrial remodeling in atrial fibrillation patients. MIP-1*α*, also known as CCL3, is a cytokine belonging to the CC chemokine family, known for its role in leukocyte activation and migration to inflammatory areas. In arrhythmic cardiomyopathy [11], chemokine expression profiles such as CCL3/CCR5 and CXCL5/CXCR2 mRNA have been verified to modulate inflammatory and repair processes throughout the progression of arrhythmic cardiomyopathy and CCL3 is a major chemokine throughout the entire disease process. Atrial fibrillation is a common arrhythmia. Taken together, understanding the MIP-1*α* level and its correlation with the risk of left atrial remodeling may provide a new direction for the diagnosis and treatment of atrial fibrillation.

In the tumor microenvironment [12], MIP-1*α* affects key factors in the migration and maintenance of relevant immune cells into infected tissues or the tumor microenvironment. When CD4 is released, CCL3+ T cells interact with dendritic cells, and CD8+ T cells expressing CCR5 were recruited to enter specific locations to activate and proliferate in living organisms. In recent years, with the deepening of the research, the MIP-1*α* effect on the tumor microenvironment has gradually transferred to cardiovascular diseases. MIP-1*α* can be utilized to predict clinical outcomes in patients with atherosclerotic cardiovascular disease, myocardial ischemia, and heart failure [13]. In cardiac-specific transgenic mice [14], the CCR9 and CCL3 overexpression enhanced pressure overload-induced cardiac hypertrophy; CCL3 and CCL4 levels were higher in the hearts of transverse aortic stenosis mice compared with sham-operated mice. This study found that compared with the normal population, serum MIP-1*α* levels were higher in patients with atrial fibrillation, indicating that MIP-1*α* was highly expressed in atrial fibrillation patients. Inflammatory response and oxidative stress exist in the occurrence of atrial fibrillation. Sustained inflammatory response and excessive oxidative stress can activate NF-KB and release MIP-1*α*. High MIP-1*α* levels can promote the electrical and structural remodeling of the heart. Therefore, MIP-1*α* is highly expressed in atrial fibrillation patients.

Left atrial enlargement is considered a marker of atrial remodeling and typically occurs in response to left atrial pressure and volume overload in patients with atrial fibrillation. A previous study [15] has demonstrated that inflammatory and fibrotic cytokines are not only associated with the occurrence of atrial fibrillation but also participate in left atrial remodeling in atrial fibrillation patients. The results from a study [16] by Sun et al. exhibited that persistent atrial fibrillation patients with pulmonary infection presented high serum inflammatory factor levels, and the increased serum inflammatory factor levels were correlated with the degree of left ventricular remodeling, suggesting that the progression of left atrial remodeling may be associated with the inflammatory response in patients with atrial fibrillation. Cytokines produced by macrophages, including interleukin (IL)-1, IL-6, and TNF-*α*, have been implicated in atrial fibrosis and episodes of atrial fibrillation [17]. In terms of atrial remodeling, Hafner et al. [18] suggested that during atrial damage caused by volume or pressure overload and inflammation, cardiac fibroblasts or cardiac macrophages may secrete MIP-1*α*, which may induce leukocyte activation and migration to inflammatory areas and participate in the repair process. It was found in MIP-1*α*-induced experimental autoimmune myocarditis [19] that MIP-1*α* plays a key role in myocardial fibrosis. Another study has confirmed that [20] MIP-1*α* can induce monocytes to produce matrix metalloproteinase 9 and TGF-*β* expression, while MMP-9 and TGF-*β* accelerate the progression of atrial fibrillation by increasing the degree of atrial fibrosis and participate in the left atrial remodeling in atrial fibrillation patients. These studies indicate that the MIP-1*α* level may be involved in the left atrial remodeling in atrial fibrillation patients. The results from the present study displayed that the anteroposterior diameter, upper and lower diameter, left and right diameter of the left atrium, left atrial volume, volume index, and sphericity were higher but the left atrial global ejection fraction was lower in the high-level group than those in the low-level group. Further correlation analysis results revealed that MIP-1*α* levels were negatively correlated with the left atrial global ejection fraction but positively correlated with the remaining left atrial remodeling indexes, indicating that MIP-1*α* can remarkably predict left atrial remodeling in patients with atrial fibrillation. This is associated with the fact that elevated MIP-1*α* levels can promote the activation and migration of leukocytes to inflammatory areas, leading to left atrial remodeling.

In conclusion, serum MIP-1*α* expression levels are high in patients with atrial fibrillation, and MIP-1*α* levels are associated with the risk of left atrial remodeling. This study has certain limitations. First, the serum MIP-1*α* expression level was not dynamically analyzed, and the correlation between dynamic serum MIP-1*α* level and the risk of left atrial remodeling could not be observed. Second, due to the limitation of objective conditions such as sample size, only the left atrial remodeling indicators were analyzed in patients with atrial fibrillation, and the electrical remodeling of the left atrium was not considered. Further investigations are needed and will make up for the abovementioned shortcomings.

## Figures and Tables

**Figure 1:** Comparison of serum MIP-1*α* levels.

**Figure 2:** Heatmap of the correlation between serum MIP-1*α* levels and the risk of left atrial remodeling in patients with atrial fibrillation.

**Table 1:** Comparison of clinical data of the case group.

Item	High-level group (*n* = 32)	Low-level group (*n* = 32)	*t*/*χ*^2^ value	*P* value
Sociodemographic data				
Age ($\bar{x}\pm s$, year)	42.96 ± 8.57	41.09 ± 9.01	0.851	0.398
Sex (male/female)	20/12	19/13	0.066	0.798
Body mass index ($\bar{x}\pm s$, kg/m^2^)	23.02 ± 1.05	23.05 ± 1.03	0.115	0.909
Atrial fibrillation course ($\bar{x}\pm s$, year)	3.85 ± 1.11	3.79 ± 1.12	0.215	0.830

Comorbidities (*n*, %)				
Hypertension	10 (31.25)	8 (25.00)	0.309	0.578
Diabetes	5 (15.63)	4 (12.50)	0.129	0.719
Hyperlipidemia	8 (25.00)	7 (21.88)	0.087	0.768
Coronary artery disease	7 (21.88)	6 (18.75)	0.097	0.756
CHA2DS2 –VASC score ($\bar{x}\pm s$, point)	3.07 ± 0.84	3.01 ± 0.78	0.296	0.768

Type of atrial fibrillation (*n*, %)			0.250	0.617
Paroxysmal	15 (46.88)	17 (53.12)		
Persistent	17 (53.12)	15 (46.88)		

New York Heart Association function classification (*n*, %)			0.251	0.616
Class I	16 (50.00)	18 (56.25)		
Class II	16 (50.00)	14 (43.75)		

**Table 2:** Comparison of left atrial remodeling indexes in the case group.

Item	High-level group (*n* = 32)	Low-level group (*n* = 32)	*t*/*χ*^2^ value	*P* value
Left atrial anteroposterior diameter ($\bar{x}\pm s$, mm)	49.99 ± 7.63	46.02 ± 8.01	2.030	0.047
Left atrial left and right diameter ($\bar{x}\pm s$, mm)	77.95 ± 9.62	72.02 ± 10.28	2.383	0.020
Left atrial upper and lower diameter ($\bar{x}\pm s$, mm)	68.85 ± 10.02	63.85 ± 9.87	2.011	0.049
Left atrial volume ($\bar{x}\pm s$, mL)	169.52 ± 40.28	147.78 ± 41.98	2.114	0.039
Left atrial volume index ($\bar{x}\pm s$, ml/m^2^)	96.25 ± 20.54	84.95 ± 19.87	2.237	0.029
Left atrial global ejection fraction ($\bar{x}\pm s$, %)	50.24 ± 4.98	53.29 ± 5.26	2.633	0.020
Left atrial sphericity ($\bar{x}\pm s$, %)	87.54 ± 7.25	83.25 ± 6.98	2.411	0.019

## Data Availability

The simulation experiment data used to support the findings of this study are available from the corresponding author upon request.
